RETRACTED

# miR-223-5p Suppresses OTX1 to Mediate Malignant Progression of Lung Squamous Cell Carcinoma Cells

**DOI:** 10.1155/2021/6248793

**Published:** 2021-07-08

**Authors:** Yunping Lu

**Affiliations:** Department of Cardio-Thoracic Surgery, Affiliated Jinhua Hospital, Zhejiang University School of Medicine, Jinhua, China

## Abstract

**Background:**

Lung squamous cell carcinoma (LUSC) features high morbidity and mortality as a worldwide malignant tumor. This study mainly explored a miR-223-5p-dependent mechanism that affected proliferation, invasion, and migration of LUSC cells.

**Methods:**

Expression data of mature miRNAs and sequencing data of total RNA of LUSC were downloaded from TCGA database. Differentially expressed mRNAs were obtained. Function of miR-223-5p in LUSC cells was detected by assays like qRT-PCR, MTT, wound healing assay, Western blot, and Transwell assay. Western blot was performed to analyze the relationship between OTX1 and JAK/STAT signaling pathways. Dual-luciferase assay detected the relationship between miR-223-5p and OTX1. The way how miR-223-5p regulated LUSC cell biological functions via OTX1 was further explored.

**Results:**

It was noted that miR-223-5p expression in LUSC tissue and cells was significantly reduced. Overexpression of miR-223-5p negatively regulated the proliferation, invasion, and migration of LUSC cells. The downstream target gene OTX1 was detected to be notably elevated in LUSC cells. A negative correlation between OTX1 and miR-223-5p was also found. As analyzed by GSEA, OTX1 was significantly enriched in the JAK/STAT signaling pathway and activated the pathway. Dual-luciferase assay demonstrated that OTX1 was a direct molecular target of miR-223-5p in LUSC cells. Rescue experiment verified that miR-223-5p regulated the malignant phenotypes of LUSC cells by pairing with OTX1.

**Conclusion:**

This study indicated that miR-223-5p was lowly expressed in LUSC cells. The impact of miR-223-5p on cell proliferation, invasion, and migration was realized by targeting OTX1. It is likely that miR-223-5p can be a novel target for LUSC treatment, which provides new ideas for future LUSC treatment.

## 1. Introduction

Being the most common malignancy in the world and the predominant cause of cancer death, lung cancer triggers a 5-year survival rate only of 19% [1]. Referring to the classification of the World Health Organization (WHO), lung cancer can be grouped into two subtypes in pathology: non-small-cell lung cancer (NSCLC) and small cell lung cancer (SCLC). Of the two types, NSCLC can be further divided into lung squamous cell carcinoma (LUSC), lung adenocarcinoma (LUAD), and large cell lung cancer (LCLC) [2]. LUSC kills about 400,000 worldwide annually since 70% of patients have progressed to an advanced stage when being diagnosed [3, 4]. Treatment approaches for LUSC mainly are surgery and radiotherapy or chemotherapy, which are inefficient for advanced patients. However, biomarker-oriented treatment is an effective approach to improving advanced LC patient's overall survival [5]. Nevertheless, recognized biomarkers for treatment of LUSC are lacking. Hence, exploring new biomarkers is imperative for improving clinical diagnosis and treatment of LUSC.

RETRACTED

MicroRNAs (miRNAs), evolutionarily conserved noncoding RNA (about 22 nucleotides), are modifiers that posttranscriptionally regulate gene expression [6]. miRNAs can reversely regulate gene expression by incomplete base pairing within the 3′ untranslated region (UTR) of targeted genes, leading to mRNA degradation [7, 8]. miRNAs can inhibit gene expression by degrading mRNA, then mediating various cell functions, including tumor cell invasion and metastasis [9]. miR-223-5p plays a part in many cancers. It is found that miR-223-5p acts as an inhibitor in the progression and lung metastasis of osteosarcoma [10]. In vulvar cancer, miR-223-5p correlates with metastasis, and overexpressing miR-223-5p suppresses the proliferation and migration of vulvar cancer cells [11]. In NSCLC, miR-223-5p can hinder tumor growth and metastasis via regulating E2F8 [12]. Nevertheless, the mechanism of miR-223-5pin LUSC requires further clarification.

Therefore, it is important to thoroughly identify the role of miR-223-5p in LUSC and clarify underlying molecular mechanisms. Here, the role and mechanism that miR-223-5p regulates the proliferation, migration, and invasion of LUSC cells were explored by a series of cellular and molecular assays. This study can provide support for further understanding the pathogenesis of LUSC.

## 2. Materials and Methods

### 2.1. Cell Culture

Normal human lung epithelial cell line BEAS-2B (3131C0001000200027) was ordered from Cell Bank of Shanghai Institutes for Biological Sciences, Chinese Academy of Sciences. LUSC cell lines H2170 (3111C0001CCC000354) and H1703 (3111C0001CCC000353) were obtained from Cell Bank of Institute of Basic Medical Sciences, Chinese Academy of Medical Sciences. LUSC cell lines SK-MES-1 (3142C0001000000946) and H226 (3142C0001000000966) were accessed from Cell Bank of China Center for Type Culture Collection (CCTCC). With a culture condition at 37°C with 5% CO_2_, all the cell lines were grown in a RPMI-1640 medium (Gibco, Rockville, MD, USA) added with 1% penicillin (Invitrogen) and 10% fetal bovine serum (FBS; Gibco).

### 2.2. Bioinformatics Analysis

Expression data of mature miRNAs (including 473 cancer tissue samples and 45 adjacent normal tissue samples) and sequencing data of RNA-seq (including 497 cancer tissue samples and 49 adjacent normal tissue samples) were obtained from TCGA-LUSC dataset (https://portal.gdc.cancer.gov/). miR-223-5p expression was differentially analyzed referring to the downloaded data. Differentially expressed mRNAs (DEmRNAs) were detected by R package “edgeR” (∣logFC | >2, *p*adj < 0.05). Target genes of miR-223-5p were researched in miRTarBase and TargetScan databases. The results were intersected with upregulated DEmRNAs, and candidate DEmRNAs which have binding sequences of miR-223-5p were screened out. The target mRNA was identified by correlation analysis.

RETRACTED

### 2.3. Cell Transfection

miR-223-5p mimics, miR-223-5p inhibitor, and NCs were ordered from Shanghai GenePharma. Small interfering RNAs (siRNAs) targeting OTX1 were made by Shanghai Sangon Biotech Co, Ltd. Recombinant plasmids pEGFP1-OTX1 were made using overexpressing vectors pEGFP1. Mimics, siRNAs, inhibitors, recombinant plasmids, and corresponding controls were taken for transfection treatment using Lipofectamine®3000 (Invitrogen, USA) following the instructions.

### 2.4. Real-Time Quantitative Polymerase Chain Reaction (qRT-PCR)

Total RNA obtained by Trizol (Invitrogen) from cells was taken to synthesize cDNA on a reverse transcription system (Promega). Expression of miR-223-5p and OTX1 mRNA was quantified with the SYBR PrimeScript miRNA RT-PCR kit (Takara, Dalian, China). cDNA templates were amplified on the ABI 7900 real-time fluorescence quantification PCR instrument (Applied Biosystems, CA, USA). qRT-PCR conditions were as below: 94°C, 3 min; 34 cycles: 94°C, 15 s; 60°C, 55 s; and 72°C, 30 s. OTX1 mRNA and miR-223-5p were internally referenced to GAPDH and U6, respectively. The results were shown with a 2^-*ΔΔ*Ct^ value. The experiment was repeated 3 times. Primer sequences are listed in Table 1.

### 2.5. Western Blot Assay

Pretreated with cold phosphate-buffered saline (PBS), transfected cells were exposed to radioimmunoprecipitation assay (RIPA) lysis buffer added with 1% protease inhibitor (Sigma-Aldrich) for protein extraction. Protein concentration was assessed with the BCA protein assay kit (Thermo Fisher Scientific, Waltham, MA, USA). Protein samples at 40 *μ*L/lane were separated by sodium dodecyl sulfate polyacrylamide gel electrophoresis (SDS-PAGE) (Bio-Rad, Hercules, CA, USA). Then, the separated proteins were transferred onto a polyvinylidene fluoride (PVDF) membrane (Millipore, Billerica, MA, USA). Following an incubation with 5% skim milk powder, the membrane was incubated overnight at 4°C using target primary antibodies, followed by 2 h of hybridization with horseradish peroxidase-labeled secondary antibody goat anti-rabbit IgG. Tris-Buffered Saline Tween-20 (TBST) (Sigma-Aldrich) was used to wash the membrane three times. Protein bands were detected with electrochemiluminescence (ECL; Beyotime, Shanghai, China), and quantitative analysis was conducted with Image Lab (Bio-Rad). The experiment was repeated 3 times. (Antibody information is shown in Table 2.)

RETRACTED

### 2.6. Cell Proliferation Assay

SK-MES-1 cells were prepared into single cell suspension with culture solution containing 10% FBS, which was inoculated into 96-well plates for 200 *μ*L per well (5 × 10^3^ cells per 100 *μ*L). Each group was treated in triplicate. MTT solution (Solarbio, M1020) (5 mg/mL with PBS) (20 *μ*L) was added into each well at indicated time points (0 h, 12 h, 24 h, 48 h, and 72 h). Cells were incubated for further 4 h. The supernatant in the wells was absorbed and abandoned. Afterwards, cells were centrifuged and the supernatant was absorbed and abandoned once again. DMSO (dimethyl sulfoxide) (150 *μ*L) was added to make crystals fully melt. A spectrophotometer (Molecular Devices, Sunnyvale, CA, USA) was applied to measure the absorbance of each well at 490 nm wavelength.

### 2.7. Wound Healing Assay

SK-MES-1 cells were seeded in 3.5 cm plates and incubated in RPMI 1640 culture medium. When the growing cell layers were confluent, a straight scratch through the center of the well on each plate was made with a sterilized pipette. PBS was used to wash the wells to remove all floating cells. Then, the cells were cultured in serum-free medium for 24 h. Wound healing was monitored and photographed at 0 h and 24 h, respectively.

### 2.8. Transwell Invasion Assay

All culture reagents and Transwell chambers were placed at 37°C. When the growth of SK-MES-1 cells reached to logarithmic phase, the cells were digested, washed with PBS, and suspended by serum-free medium successively. Cell concentration was adjusted to 2 × 10^5^ cells/mL. The lower chambers were filled with culture medium (600-800 *μ*L) with 10% serum while the upper chambers were added with 100-150 *μ*L of cell suspension. The upper chambers were covered with Matrigel. Following 24 h of incubation, the chambers were moved out with forceps. Liquid in upper chambers was drained. The chambers were transferred to a plate which was prefilled with about 800 *μ*L of methanol per well. After fixation at room temperature for 30 min, the chambers were moved out and the liquid in upper chambers was drained. The cells on the upper surface of the membrane were wiped off with a cotton swab applicator. The membrane was removed with small forceps, and cells under the membrane were dyed with 0.5% crystal violet. Then, the dyed cells were observed under a microscope.

RETRACTED

### 2.9. Dual-Luciferase Reporter Gene Assay

Wild-type (WT) and mutant (MUT) 3′ UTR of OTX1 were linked to the downstream of the luciferase reporter gene in target vectors. Luciferase plasmids OTX1-WT and OTX1-MUT were constructed. Afterwards, mimic-NC and miR-223-5p mimic were cotransfected to SK-MES-1 cells with OTX1-WT and OTX1-MUT, respectively. With the Renilla luciferase vector pRL-TK (TaKaRa, Dalian, China) as the internal reference, luciferase activity was measured with luciferase reporter gene assay kits.

### 2.10. Statistics

Prism 8.0 was used for data processing. Mean ± standard deviation was applied to show measurement data, and *t*-test was used to analyze the difference between two groups. *p* < 0.05 was set as a threshold to define statistical significance.

## 3. Results

### 3.1. Decreased Expression of miR-223-5p in LUSC Cell Lines and Tissue

Expression data of mature miRNA and RNA sequencing data obtained from TCGA-LUSC dataset were used to analyze the expression of miR-223-5p in LUSC. miR-223-5p was found to be notably poorly expressed in LUSC (Figure 1(a)). As reported, overexpressed miR-223-5p could make an effect on cell proliferation, migration, and invasion of NSCLC as a tumor suppressor [12]. In this study, miR-223-5p expression in LUSC cell lines H2170, H1703, SK-MES-1, and H226 was analyzed by qRT-PCR. Markedly decreased miR-223-5p expression in these cell lines was noted than that in human normal cell line BEAS-2B (Figure 1(b)). Of these cancer cell lines, miR-223-5p expression in SK-MES-1 cell line was the lowest. Therefore, SK-MES-1 was chosen for further experiments. The results of these experiments showed that miR-223-5p expression was reduced in LUSC cell lines and tissue.

### 3.2. miR-223-5p Inhibits Malignant Behaviors of LUSC Cells *In Vitro*

In order to explore how miR-223-5p affects the proliferation, invasion, and migration of LUSC cells, miR-223-5p mimic/inhibitor and their control mimic/inhibitor were, respectively, transfected into LUSC cell line SK-MES-1. The result of qRT-PCR revealed that miR-223-5p mimic significantly increased miR-223-5p expression in SK-MES-1, while miR-223-5p inhibitor decreased miR-223-5p expression (Figure 2(a)). Then, how overexpression or inhibition of miR-223-5p affected LUSC cell proliferation, invasion, and migration was detected by a series of assays including MTT assay, Transwell assay, and wound healing assay. The results demonstrated that compared with the corresponding control group, overexpressing miR-223-5p highly suppressed SK-MES-1 cell activities in proliferation, invasion, and migration, while silenced miR-223-5p promoted such abilities (Figures 2(b)–2(d)). It indicated that miR-223-5p inhibited the *in vitro* proliferation, invasion, and migration of LUSC cells.

RETRACTED

### 3.3. miR-223-5p Binds to OTX1 and Inhibits OTX1 Expression

To gain more insight into the regulatory mechanism of miR-223-5p in LUSC, R package edgeR was used for differential expression analysis (∣logFC | >2, *p*adj < 0.05). 3,469 DEmRNAs were obtained in the TCGA-LUSC, of which 1,179 were downregulated and 2,290 were upregulated (Figure 3(a)). The upregulated DEmRNAs were intersected with the targeted genes of miR-223-5p predicted by TargetScan and miRTarBase databases. 19 candidate targeted genes were obtained (Figure 3(b)), of which OTX1 was significantly highly expressed in cancer LUSC tissue (Figure 3(c)). OTX1 had the strongest negative correlation with miR-223-5p according to correlation analysis (Figure 3(d)). OTX1 is reported to have the ability of promoting the proliferation and metastasis of hepatocellular carcinoma and colorectal cancer [13, 14]. Hence, OTX1 was chosen as a possible target of miR-223-5p for further study. Potential binding sites between miR-223-5p and OTX1 were predicted by miRTarBase database (Figure 3(e)). In addition, the binding sites between these two genes were mutated and dual-luciferase assay was used to identify the validity of the binding sequence. The result showed that overexpressed miR-223-5p significantly lowered the luciferase activity of cells with OTX1-WT, with no effect on OTX1-MUT (Figure 3(f)). The results of qRT-PCR and Western blot showed that overexpressing miR-223-5p could inhibit OTX1 mRNA and protein expression, while inhibition of miR-223-5p could promote OTX1 expression (Figures 3(g) and 3(h)). These assays indicated that miR-223-5p inhibited OTX1 expression.

### 3.4. OTX1 Induces JAK/STAT Signaling Activation and Promotes the Proliferation, Invasion, and Migration of LUSC Cells

OTX1 was subjected to GSEA, and the result showed that OTX1 was significantly activated in the JAK/STAT signaling pathway (Figure 4(a)). It is known that the JAK/STAT signaling pathway can promote tumor cell survival, proliferation, and invasion [15]. Therefore, we further explored whether OTX1 could regulate the JAK/STAT signaling pathway. Here, we examined the expression of proteins relevant to the JAK/STAT pathway in LUSC cells SK-MES-1 transfected with oe-OTX1 and si-OTX1. It was found that overexpressed OTX1 could promote phosphorylation of STAT5 and JAK2 in SK-MES-1 by Western blot, while silenced OTX1 could inhibit the phosphorylation. However, total protein expression of STAT5 and JAK2 was not significantly affected (Figure 4(b)). To identify the influence of OTX1 on LUSC cells, qRT-PCR was used to detect transfection efficiency (Figure 4(c)). MTT assay was used to determine the role of overexpressed OTX1 or silenced OTX1 in SK-MES-1 proliferation. As analyzed, overexpressed OTX1 greatly increased SK-MES-1 proliferation while silenced OTX1 inhibited such ability (Figure 4(d)). The results of Transwell assay showed that overexpressed OTX1 could significantly promote SK-MES-1 invasion while silenced OTX1 could significantly inhibit the ability (Figure 4(e)). As revealed by wound healing assay, silenced OTX1 could markedly reduce SK-MES-1 migration while overexpressed OTX1 could enhance the migrative ability (Figure 4(f)). These assays demonstrated that OTX1 could activate the JAK/STAT signaling pathway and thus elevate the proliferative, migratory, and invasive abilities of LUSC cells.

RETRACTED

### 3.5. miR-223-5p Suppresses Biological Behaviors of LUSC Cells by Targeting OTX1

To further elucidate the miR-223-5p-dependent molecular mechanism by targeting OTX1 to mediate LUSC cell biological behaviors, OTX1 overexpression vectors and miR-223-5p mimics were cotransfected into SK-MES-1 cells to detect the changes in cell proliferative, invasive, and migratory abilities. The results of qRT-PCR showed that overexpressed miR-223-5p decreased OTX1 expression, while oe-OTX1 increased the expression of OTX1. Cotransfection of miR-223-3p mimic and oe-OTX1 reversed the inhibitory effect of miR-223-5p mimic on OTX1 expression. (Figure 5(a)). The results of MTT assay showed that compared to the NC group, miR-223-3p mimic inhibited the proliferation of SK-MES-1 cells, while oe-OTX1 promoted the proliferation. Overexpressing OTX1 could reverse the inhibition of miR-223-5p on SK-MES-1 cell proliferative ability (Figure 5(b)). Transwell assay and wound healing assay were performed, and it was indicated that miR-223-3p mimic inhibited the invasion and migration of SK-MES-1 cells compared to the NC group, while oe-OTX1 promoted these functions. OTX1 could greatly reverse the inhibition of miR-223-5p overexpression on SK-MES-1 cell invasion and migration (Figures 5(c) and 5(d)). As revealed by WB assay, miR-223-5p mimic constrained the phosphorylation of STAT5 and JAK2 in SK-MES-1 cells, while oe-OTX1 stimulated the phosphorylation. However, cotransfection of miR-223-3p mimic and oe-OTX1 reversed the inhibition of miR-223-3p mimic on the phosphorylation of STAT5 and JAK2 (Figure 5(e)). These assays identified that miR-223-5p inhibited the proliferative, invasive, and migratory capabilities of LUSC cells by inhibiting OTX1 expression.

RETRACTED

## 4. Discussion

LUSC can be divided into basaloid squamous cell carcinoma (BSCC), keratinized squamous cell carcinoma (KSCC), and nonkeratinized squamous cell carcinoma (NKSCC), and it is one of the most common histological subtypes of lung cancers [16]. In the past decades, scholars have been exploring the biological function of miRNAs. More and more evidence indicates that miRNAs are vital players in various biological processes, signifying that miRNA expression is closely related to human cancers [17]. Some studies indicated that miRNAs are promising therapeutic targets for cancer interventional treatment [18]. Thus, study on miRNA is of great clinical significance. Here, the role and underlying mechanism of miR-223-5p that is involved in LUSC progression were discussed. As an important miRNA, miR-223-5p can regulate many cancers, such as gastric cancer and bladder cancer [19, 20]. Moreover, it is proven that overexpressing miR-223-5p in specific cancers can lead to unfavorable prognosis [21]. However, no research has been reported about the role of miR-223-5p in LUSC. In this study, we analyzed miRNA expression profile in TCGA-LUSC and discovered decreased miR-223-5p in LUSC. Additionally, we noted that miR-223-5p expression was associated with LUSC cell biological behaviors, including proliferation, migration, and invasion, which signified the link of miR-223-5p expression to LUSC progression for the first time. However, the effect of miR-223-5p in cancers remains disputed. The regulation of miR-223-5p on proliferation and differentiation of cancer cells may be tissue-specific. The specificity is strong which may be caused by pure *in vitro* experiments in our study. Hence, the effect of miR-223-5p awaits to be further researched. Then, we predicted the downstream gene of miR-223-5p and found that miR-223-5p could regulate OTX1 expression by binding to OTX1. As reported, OTX1 can promote colorectal cancer progression by inducing epithelial-mesenchymal transition [14]. It is also found that OTX1 actively functions on the proliferative, migratory, and invasive capabilities of gastric cancer cells [22]. In addition, OTX1 can regulate cell proliferation and migration of breast cancer via mediating ADPGK-AS1. These findings are consistent with the finding of this study that OTX1 promotes cancer progression.

Later, pathway enrichment analysis was adopted for OTX1 and it was found that OTX1 was mainly enriched in the JAK/STAT signaling pathway, which is closely connected with progression of many cancers. For example, in colorectal cancer, knockdown of TfR1 facilitates cancer progression via the JAK/STAT pathway [23]. Additionally, miR-196a/-196b can promote liver cancer progression by targeting SOCS2 and regulating JAK/STAT [24]. These studies demonstrate that phosphorylation of JAK and STAT can promote cancer progression. In this study, we found that overexpressing OTX1 could regulate cancer progression by inducing the phosphorylation of related proteins to activate the JAK/STAT pathway. Thus, we found a regulatory axis composed of miR-223-5p/OTX1/JAK/STAT. Then, to validate that miR-223-5p could mediate the proliferation, invasion, and migration of LUSC cells by downregulating OTX1, rescue experiments were conducted. The results showed that OTX1 upon overexpression could attenuate the effects of upregulated miR-223-5p on biological functions of LUSC cells.

RETRACTED

In conclusion, it was found in the present study that miR-223-5p was lowly expressed in LUSC cells and negatively functioned on the proliferative, invasive, and migratory abilities of LUSC cells. The downstream target gene OTX1 was highly expressed in cancer cells and correlated with the activation of the JAK/STAT signaling pathway. Moreover, the effect of miR-223-5p on the biological functions of LUSC cells was achieved by targeting OTX1. These results may provide reference and support for identification of new targeted therapies for LUSC. In the future, we will continue to explore the mechanism of miR-223-5p/OTX1 in LUSC *in vivo*.

## Figures and Tables

**Figure 1:** Decreased miR-223-5p in LUSC cell lines and tissue. (a) Box plots show miR-223-5p expression in TCGA-LUSC dataset; (b) miR-223-5p expression in different LUSC cell lines H2170, H1703, SK-MES-1, and H226 and one normal human lung epithelial cell line BEAS-2B was detected by qRT-PCR; ∗ means *p* < 0.05 compared to BEAS-2B.

**Figure 2:** miR-223-5p inhibits the proliferation, invasion, and migration of LUSC cells *in vitro*: (a) miR-223-5p expression in groups with miR-223-5p mimic/inhibitor detected by qRT-PCR; (b) proliferative ability of SK-MES-1 cells after miR-223-5p was overexpressed or inhibited was detected by MTT; (c) invasive ability of SK-MES-1 after miR-223-5p was overexpressed or inhibited was detected by Transwell assay (×100); (d) migratory ability of SK-MES-1 after miR-223-5p was overexpressed or inhibited was detected by wound healing assay (×40); ∗ means *p* < 0.05 while miR-223-5p mimic versus mimic-NC or miR-223-5p inhibitor versus inhibitor-NC.

**Figure 3:** miR-223-5p targets and inhibits OTX1 expression: (a) volcano plot of DEmRNAs in TCGA-LUSC; (b) intersection between targeted genes of miR-223-5p predicted by TargetScan and miRTarBase databases and the upregulated DEmRNAs in TCGA-LUSC dataset; (c) box plot of OTX1 expression in tumor and normal samples in TCGA; (d) correlation between miR-223-5p and 19 candidate targeted genes; (e) predicted binding sites between miR-223-5p and OTX1; (f) the targeted binding between miR-223-5p and OTX1 was identified by dual-luciferase assay; (g) OTX1 mRNA expression in cells overexpressing miR-223-5p or inhibiting miR-223-5p was detected by qRT-PCR; (h) OTX1 protein expression in cells overexpressing miR-223-5p or inhibiting miR-223-5p was assessed by Western blot; ∗compare miR-223-5p mimic+OTX1-WT with mimic-NC+OTX1-WT, compare miR-223-5p mimic with mimic NC, and compare miR-223-5p inhibitor with inhibitor NC, *p* < 0.05.

RETRACTED

**Figure 4:** OTX1 induces JAK/STAT signaling pathway activation and potentiates the proliferation, invasion, and migration of LUSC cells. (a) The signaling pathway regulated by OTX1 was analyzed via GSEA. (b) Relative expression of the proteins relevant to the JAK/STAT signaling pathway after OTX1 was overexpressed or silenced was detected by Western blot. (c) OTX1 mRNA expression in SK-MES-1 after OTX1 was overexpressed or silenced. (d) Changes of SK-MES-1 cell proliferation upon overexpression or silencing of OTX1 were detected by MTT assay. (e) Changes of SK-MES-1 cell invasion upon overexpression or silencing of OTX1 were detected by Transwell (×100). (f) Changes of SK-MES-1 cell migration upon overexpression or silencing of OTX1 were detected by wound healing assay (×40); ∗ means *p* < 0.05 as the oe-OTX1 group versus oe-NC, or si-OTX1 versus si-NC.

**Figure 5:** miR-223-5p inhibits the proliferation, invasion, and migration of LUSC cells by targeted inhibiting OTX1 expression: (a) changes in OTX1 mRNA expression in groups of SK-MES-1 cells with oe-OTX1 and miR-223-5p mimic detected by qRT-PCR; (b) changes in cell proliferative activity in each group detected by MTT assay; (c) changes in cell invasive potential in diverse treatment groups detected via Transwell assay (×100); (d) changes in cell migratory capability after transfection detected by wound healing assay (×40); (e) Western blot detected changes of the expression of JAK-STAT signaling pathway in each treatment group; ∗ means *p* < 0.05 between the two groups as drawn in figures.

**Table 1:** Primer sequence used in qRT-PCR.

Genes	Primer sequence
miR-223-5p	F: 5′-TGGATCCGTGTCACTCGGGCTTTACCTG-3′
	R: 5′-CGAATTCGTAGACACAGCCCAGGGCTGT-3′
GAPDH	F: 5′-GGGAGCCAAAAGGGTCATCATCTC-3′
	R: 5′-CCATGCCAGTGAGCTTCCCGTTC-3′
U6	F: 5′-CTCGCTTCGGGCAGCACA-3′
	R: 5′-AACGCTTCACGAATTTGCGT-3′
OTX1	F: 5′-GCGTCGTCGCTGAGTACAC-3′
	R: 5′-ACATGGGATAAGAGGCTGCTG-3′

**Table 2:** Antibodies used in Western blot.

Antibody	WB	Specificity	Company
*β*-Actin	1 : 5000	Rabbit monoclonal	Abcam, China
OTX1	0.5-4 *μ*g/mL	Rabbit polyclonal	Abcam, China
IgG	1 : 5000	Goat anti rabbit	Abcam, China
STAT5	0.5-4 *μ*g/mL	Rabbit monoclonal	Abcam, China
p-STAT5	0.5-4 *μ*g/mL	Rabbit monoclonal	Abcam, China
JAK2	0.5-4 *μ*g/mL	Rabbit monoclonal	Abcam, China
P-JAK2	0.5-4 *μ*g/mL	Rabbit monoclonal	Abcam, China

RETRACTED

## Data Availability

The data and materials in the current study are available from the corresponding author on reasonable request.
